The article "Passive Fetal Movement Signal Detection System Based on Intelligent Sensing Technology" was published in 2021. Journal: J Healthc Eng.

# Passive Fetal Movement Signal Detection System Based on Intelligent Sensing Technology

**DOI:** 10.1155/2021/1745292

**Published:** 2021-08-25

**Authors:** Sensong Liang, Jiansheng Peng, Yong Xu

**Affiliations:** ^1^Department of Electronic Engineering, Guangxi Normal University, Guilin, China; ^2^Department of Artificial Intelligence and Manufacturing, Hechi University, Hechi, China

## Abstract

Fetal movement (FM) is an essential physiological parameter to determine the health status of the fetus. To address the problems of harrowing FM signal extraction and the low recognition rate of traditional machine learning classifiers in FM signal detection, this paper develops a passive FM signal detection system based on intelligent sensing technology. FM signals are obtained from the abdomen of the pregnant woman by using accelerometers. The FM signals are extracted and identified according to the clinical nature of the features hidden in the amplitude and waveform of the FM signals that fluctuate in duration. The system consists of four main stages: (i) FM signal preprocessing, (ii) maternal artifact signal preidentification, (iii) FM signal identification, and (iv) FM classification. Firstly, Kalman filtering is used to reconstruct the FM signal in a continuous low-amplitude noise background. Secondly, the maternal artifact signal is identified using an amplitude threshold algorithm. Then, an innovative dictionary learning algorithm is used to construct a dictionary of FM features, and orthogonal matching pursuit and adaptive filtering algorithms are used to identify the FM signals, respectively. Finally, mask fusion classification is performed based on the multiaxis recognition results. Experiments are conducted to evaluate the performance of the proposed FM detection system using publicly available and self-built accelerated FM datasets. The classification results showed that the orthogonal matching pursuit algorithm was more effective than the adaptive filtering algorithm in identifying FM signals, with a positive prediction value of 89.74%. The proposed FM detection system has great potential and promise for wearable FM health monitoring.

## 1. Introduction

Stillbirth is a widespread problem of the world today. It is estimated that, in high-income countries, 2.6 million babies died in uteri in 2015, with one in every 113～769 pregnancies dying in utero after 28 weeks of gestation [1]. It has been suggested that active maternal perception of intrauterine FM is an economical and convenient method for the early detection of fetal impairment [2, 3]. However, most pregnant women are unaware of the health status of the fetus in their womb between pregnancy and delivery. Some fetuses are at risk of developing complications that may result in future disease, handicap, or death [4]. For those at advanced maternal age and risk, FM detection can identify those complications that potentially alter the outcome of labor and help the practitioner to make timely interventions to avoid the development of stillbirth [5]. In a population-based study in Japan, the maternal response was prolonged following reduced FM in stillbirth [6]. In some cases of stillbirth in pregnancy, more than 50% of pregnant women felt a gradual decrease in intrauterine FM in the days before the onset of stillbirth [7]. Studies have shown that the number of intrauterine movements towards a pregnant woman can last for days or even weeks from decreasing to disappearing, and doctor interventions during this period may result in a healthy, living baby [8–10]. Therefore, early detection of potential risk factors and timely intervention to reduce the likelihood of stillbirth can be achieved by establishing antenatal FM detection.

The article "Passive Fetal Movement Signal Detection System Based on Intelligent Sensing Technology" was published in 2021. Journal: J Healthc Eng.

The main clinical methods of identifying FM are ultrasound techniques and maternal perception of FM. Ultrasound technology allows visual assessment of fetal health, including intrauterine growth, amniotic fluid volume, and Doppler flow [11], but this technique requires experienced clinicians to operate the ultrasound equipment, and in addition, prolonged exposure to the intrauterine fetus to ultrasound can cause radiation damages. Another active method of identification, the self-counting of FM by the pregnant woman in a calm and stable state, is a preliminary assessment of the intrauterine health of the fetus, which, compared to ultrasound techniques, can be performed at home and is economical and convenient for monitoring the fetus during pregnancy. However, the sensitivity of FM varies greatly from pregnant women [12], and it is challenging to monitor FM in the long term by subjective judgment. In recent years, wearable health monitoring devices had become a hot spot of research in the biomedical field, and the use of wearable acceleration sensors and modern digital signal processing techniques to achieve automatic recognition of FM has received widespread attention from researchers from all walks of life [13–24]. The accelerometers are small, inexpensive, noninvasive, sensitive, and stable and have become the ideal solution for noninvasive FM recognition.

In the current field of wearable sensor-based FM signal detection measurements, some researchers use amplitude threshold-based algorithms to identify FM signals in a continuous low-amplitude noise background, provided that the pregnant woman needs to remain stable during the measurement of FM [13, 14, 16]. However, this method is susceptible to noisy signals and therefore does not achieve the desired recognition results. In some other studies, feature extraction of the raw acceleration signal was performed to obtain clinically essential features of the FM signal. The related methods include time-domain feature statistics [20] and time-frequency (TF) feature analysis [15, 18, 19]. Boashash et al. [18] proposed a TF matched pursuit (TFMP) algorithm and a TF matched filtering (TFMF) algorithm to classify and detect the FM signals recorded by accelerometers. The proposed TFMP and TFMF methods achieve positive prediction values of 83% and 85% for FM signal classification results, respectively. The automatic matching detection of FM signals was achieved with higher reliability than the amplitude threshold algorithm. However, the inability to build robust dictionary atoms, limited by human empirical observation, prevents the TFMP algorithm from rapidly decomposing the energy of the signal to below 70% during a limited number of matching iterations, resulting in missed recognition of some noise-contaminated FM signals. In addition, some researchers have used traditional machine learning classifiers to train and predict the extracted raw acceleration time- and frequency-domain feature signals that aim to distinguish the FM signal class of other noisy signal classes [17, 21–24]. Vullings and Mischi [17] proposed a method of noninvasive monitoring of FM by using TF characteristics. The support vector machine (SVM) classifier was used to train and predict the preprocessed fetal movement TF features, achieving an accuracy of 75% and a specificity of 87% for FM signal classification. The final judgment output of this method depends on a small number of support vector feature samples, and a large number of redundant sample sizes are excluded, which improves the efficiency of FM recognition. However, the algorithm is more sensitive to the kernel function and the related parameter selection, and the parameter selection is taken empirically, which is not very reliable. Zhao et al. [24] proposed a wearable system for home and long-term FM assessment. Firstly, the FM time-domain and wavelet-domain signal features of the original acceleration acquisition are extracted, then the feature sequences are downscaled using the random forest algorithm, and finally, based on the extracted features, the fuzzy ARTMAP, a lightweight machine learning algorithm, is used to classify and recognize the FM signals. The specificity of this method of FM signal classification is 99%, but the sensitivity is only 77%.

The article "Passive Fetal Movement Signal Detection System Based on Intelligent Sensing Technology" was published in 2021. Journal: J Healthc Eng.

According to the above analysis, to solve the problems of harrowing FM signal extraction and low recognition rate, this paper proposes a passive FM detection system based on intelligent sensing technology. Firstly, a Kalman filtering algorithm is used to reconstruct the FM signal containing a large amount of unpredictable random noise. Secondly, the maternal artifact signal is identified using an amplitude threshold algorithm, such as maternal body movement, breathing, and laughter being misidentified as FM signals. Finally, the *K*-singular value decomposition (K-SVD) [25] dictionary learning algorithm was used to build a complete dictionary of FM and non-FM features, and the orthogonal matching pursuit (OMP) and adaptive filtering algorithms [26] were used to achieve automatic recognition of FM signals, respectively. The experimental results validate the strong robustness of the method of FM signal detection and improve the reliability and accuracy of FM detection. The main contributions to this paper are as follows:

- The K-SVD dictionary learning algorithm is proposed to obtain a complete dictionary of FM features of the training of a large number of FM datasets, which compensates for the shortcomings of constructing dictionary atoms by human empirical observation. The accuracy of recognition is improved. The Kalman filter is used to reconstruct the FM signal in a continuous low-amplitude noise background. Both improve the denoising performance of the system and reduce the complexity of the computation. At the same time, the performance of the proposed orthogonal matching pursuit algorithm and the adaptive filtering algorithm are compared for FM signal detection.
- The FM signal acquisition and recognition system uses a miniature ultralow-power processor and accelerometers. It increases the endurance of the system and also facilitates integration into a soft wearable circuit board. The microprocessor has an on-chip-integrated low-power Bluetooth communication module, which allows the data returned by the front-end sensor to be uploaded in real time via a wireless communication protocol and the data to be received and saved on the smartphone APP side. The current FM status is observed through data visualization.
- The wearable FM detection system proposed in this paper can quickly detect fluctuating signals in the abdomen of pregnant women and identify *M* signals using dictionary-based learning and sparse representation algorithms, which can meet the FM monitoring needs of pregnant women during pregnancy. The system has significant medical value in the field of e-health.

## 2. Materials and Methods

The proposed FM detection system consists of four key components: (1) FM signal preprocessing, (2) artifact signal identification, (3) FM signal identification, and (4) FM classification. The block diagram of the flow of the proposed FM detection system is shown in Figure 1. The specific description is as follows:

- FM signal preprocessing is preprocessing of the maternal abdominal wall fluctuation signals collected from each of the six axes of the dual acceleration sensors using the Kalman filter algorithm
- The artifact signal identification is performed on the preprocessed signal using an amplitude threshold algorithm to identify whether it contains maternal feature artifacts
- The K-SVD dictionary learning algorithm is used to build a complete dictionary of FM and non-FM features, and the OMP and adaptive filtering algorithms are used to match the features of the preidentified signals, respectively, and the label corresponding to the dictionary with the most minor reconstruction error is used as the recognition result
- The recognition results of the six axes are judged according to the mask fuser Mk (1 : 6) as the final classification output of the system

The article "Passive Fetal Movement Signal Detection System Based on Intelligent Sensing Technology" was published in 2021. Journal: J Healthc Eng.

### 2.1. Preprocessing of the FM Signal

The FM signal is preprocessed using the Kalman filtering algorithm. A sliding window needs to be added to the signal before preprocessing. Studies have shown that the FM signal is divided into single- and double-crested movements and is distributed over a range of 2.56 s with a sampling frequency of 100 Hz. Therefore, the time window used in this paper is 2.56 seconds, with no overlap between windows. The acceleration sensor is susceptible to the effects of external noise and other factors, mainly DC components and random noise. The DC component can be corrected simply by the equation Δ*S*=*Sk* − *Sk* − 1, *k*=1,2,3,…, *n*, where Δ*S* represents the amount of signal change from one moment to the next. However, the random noise from artefactual signals such as maternal breathing, coughing, laughter, and body movement is unpredictable and cannot be corrected by simply calculating the amount of change using the above method and requires a filter to eliminate the random noise. To process random signals, the Kalman filter is optimal and most efficient. Therefore, the Kalman filtering algorithm is used for the preprocessing of the FM signal in this paper.

The Kalman filter principle uses the previous moment's estimate and the current moment's observation to make an optimal estimate of the system state at the present moment. The equation of state is shown as follows:

(1) $$\begin{array}{c} x_{k}=A_{k}x_{\left(k-1\right)}+B_{k}u_{k}+w_{k}, \end{array}$$

where *A*_*k*_ is the state transfer matrix, *B*_*k*_ is the input matrix of the system, *u*_*k*_ is the system input at moment *k*, and *w*_*k*_ is the system process noise. If the system has no input matrix, initialize *B*_*k∗*_*u*_*k*_ to 0. According to the equation of state, the measured values are obtained as follows:

(2) $$\begin{array}{c} y_{k}=H_{k}x_{k}+V_{k}, \end{array}$$

where *H*_*k*_ is the system measurement matrix and *V*_*k*_ is the system measurement noise. In the general model, *w*_*k*_ and *V*_*k*_ are set to obey a Gaussian distribution.

The article "Passive Fetal Movement Signal Detection System Based on Intelligent Sensing Technology" was published in 2021. Journal: J Healthc Eng.

The Kalman filtering algorithm works in two stages: prediction and update. The specific steps of the Kalman filtering algorithm for the preprocessing of FM signals are given in Algorithm 1.

According to the Kalman filtering algorithm, the FM signals before and after reconstruction are obtained, as shown in Figure 2.

### 2.2. Artifact Signal Detection

The purpose of artifact recognition is to identify artifacts such as movement of the pregnant mother's body or artifacts such as heartbeat, laughter, and coughing to avoid these signals being misidentified as FM signals. Usually, the peak amplitude of artifact signals such as maternal body movement, laughter, and coughing is more significant than 0.1 g, the peak amplitude of respiratory signals is less than 0.015 g, and the peak amplitude of other background noise signals is between 0.06 g and 0.1 g, while the peak amplitude of FM signals is roughly distributed between 0.015 g and 0.06 g. These parameters are obtained from empirical observations of FM signals, background noise, and non-FM signals recorded by typical accelerometers [19]. The maternal body position movement created the artefactual noise signal fragment shown in Figure 3. Based on the above analysis, the lower limit of the amplitude threshold for the amplitude threshold prerecognition algorithm in this paper is *A*1 = 0.015 g, and the upper limit is *A*2 = 0.06 g, and the peak amplitude of the preprocessed signal fragment is within this range before it can enter the detector. The signals are collected by the two acceleration sensors within each time window set; if one of the sensors has an axis signal with a peak amplitude greater than *A*3 = 0.1 g, then the signal is identified as a characteristic artifact and classified as non-FM, ending this identification. If the peak signal amplitude is more excellent than 0.015 g and less than 0.06 g, then the current signal fragment can proceed to the next level of the detector. If the peak signal amplitude of an axis is more significant than 0.06 g and less than 0.1 or less than 0.015 g, then no feature artifacts are identified, and a binary zero is output to the mask fuser, which is combined with the signal identification results of the other axes to form the final production.

The article "Passive Fetal Movement Signal Detection System Based on Intelligent Sensing Technology" was published in 2021. Journal: J Healthc Eng.

### 2.3. FM Signal Detection

#### 2.3.1. Feature Dictionary Learning

Dictionary learning filters out the redundant noise of the signal and captures its essential features. In this paper, the K-SVD algorithm is used to learn the FM training set *Y*1 and the non-FM training set *Y*2 to construct a complete FM signal dictionary *D*1 and a non-FM signal dictionary *D*2, respectively, and the problem can be expressed as

(3) $$\begin{array}{c} \underset{D,X}{\min}Y-DX_{F}^{2},\\ \text{s.t.}\forall i.x_{i}\leq T_{0}, \end{array}$$

where *Y*=[*y*_1_, *y*_2_,…, *y*_*L*_] ∈ *R*^*m*×*L*^ denotes the training sample matrix, and each column is a training sample. *L* is the number of training samples. *D* ∈ *R*^*m*×*n*^ indicates a dictionary to be studied. *X* = [*x*_1_, *x*_2_,…, *x*_*L*_] ∈ *R*^*n*×*L*^ denotes a matrix composed of sparse coefficients.

Equation (3) is more challenging to calculate optimally for both the dictionary *D* and the sparse coefficient *X*. K-SVD uses an iterative approach to its alternate optimization. The algorithm consists of three main stages: the first stage is the initialization of the dictionary; the second stage is the sparse encoding stage, where *L* training samples in the training set *Y* are sparsely decomposed in turn using the OMP algorithm; the third stage, the dictionary update stage, uses the singular value decomposition algorithm to decompose the sparse coefficients and the dictionary according to the error minimization principle, continuously approaching the error minimization until the dictionary and the sparse coefficient matrix are obtained. The feature dictionary constructed using the K-SVD dictionary learning algorithm is shown in Figure 4. The length of the fetal and nonfetal dictionaries is 256*∗*256, respectively, which are complete dictionaries.

#### 2.3.2. FM Signal Sparse Detection

A complete feature dictionary is constructed from the above K-SVD dictionary learning. The OMP algorithm is used to match the feature atoms in the dictionary with the FM signal samples to achieve an optimal linear approximation of the FM signal samples. According to the sparsity coefficient, the reconstruction error of the FM signal samples on the FM and non-FM feature labels, respectively, is calculated. The class with the lowest reconstruction error is selected as the label for this FM signal sample, thus achieving sparse recognition. The specific steps for the identification of light FM signals are shown in Algorithm 2.

#### 2.3.3. Adaptive Filtering Detection of FM Signals

The adaptive least mean square (LMS) algorithm is an application of Wiener filtering. Each tap weight of the filter is optimized iteratively to minimize the mean square error between the original and reference signals [27]. The steps of the LMS algorithm are as follows:

(a) Compute an FIR filter system $\hat{r}\left(n\right)$ with a causal sequence that can be approximated by a finite-length *M* point sequence. This is shown in the following equation:
  (4) $$\begin{array}{c} \hat{r}\left(n\right)=\sum_{m=0}^{M}w_{m}\left(n\right)r\left(n-m\right), \end{array}$$
where *M* denotes the order of the filter.
(b) Calculate the instantaneous error *e*(*n*) at the current moment. This is shown in the following equation:
  (5) $$\begin{array}{c} e\left(n\right)=d\left(n\right)-\hat{r}\left(n\right). \end{array}$$
(c) Update the filter weights *w*_*m*_(*n*) using a recursive approach. This is shown in the following equation:
  (6) $$\begin{array}{c} w_{m}\left(n+1\right)=w_{m}\left(n\right)+2\mu e\left(n\right)r\left(n-m\right),\;\text{for }0<m<M. \end{array}$$
(d) *n*=*n*+1. Repeat the above steps until the condition is met and stop iterating.

The FM signals are detected using an adaptive filtering algorithm, and the reference signals are obtained using dictionaries *D*1 and *D*2 obtained from dictionary learning described above, with *D*1 representing the FM class and *D*2 representing the non-FM class. The optimal linear approximation of the test samples is achieved by adaptively traversing the feature atoms in both dictionaries and matching the test samples. According to the optimal filtering output and the mean square error value of the test sample, the class corresponding to the feature atom with the smallest error is selected as the class label of this test sample, and the identification of the FM signal is achieved.

The article "Passive Fetal Movement Signal Detection System Based on Intelligent Sensing Technology" was published in 2021. Journal: J Healthc Eng.

### 2.4. FM Classification

This stage classifies FM based on the mask-fused binary vector Mk (1 : 6), where binary 1 indicates an FM signal and 0 indicates a non-FM signal. If the signal from one or more axes of each of the two accelerometers is identified as an FM signal, the output of the mask fusion results in one and is classified as an FM. Otherwise, it is classified as a non-FM. A flowchart of the mask fusion process is shown in Figure 5.

## 3. Datasets and Evaluation Indicators

### 3.1. Datasets

The data sources used in this paper are a self-designed FM signal acquisition system and FM acceleration data from the Zenodo public database (ZFMAD) [28].

To verify the performance of the FM detection system proposed in this paper, the FM signal acquisition and the FM recognition experiments based on the OMP algorithm shown in Figure 6 were carried out. An acceleration sensor is designed on each side of the leading hardware circuit board to detect FM signals. The hardware circuit system consists of two 3-axis acceleration sensors (mCube, MC3672), a 32 bit microprocessor (Nordic, nRF52840), and an on-chip low-power Bluetooth module. The on-chip wireless Bluetooth communication protocol on the controller uploads the data collected by the front-end accelerometer to the mobile app for storage and visualization. For ease of transmission, the raw data collected by the two acceleration sensors were experimentally amplified by a factor of 10,000 before being uploaded. The main circuit board containing the accelerometer and microprocessor is packaged in a portable case along with a lithium battery, and a belt is used to secure the device to the pregnant woman's abdomen to ensure stable measurements over time. The measurement range of the acceleration sensor is set to ±2*g* (1*g* = 9.8 m/s^2^), the sensitivity is 4096 times/g, and the sampling frequency is set to 100 Hz. The I2C protocol is used for transmission between the sensor and the processor.

The article "Passive Fetal Movement Signal Detection System Based on Intelligent Sensing Technology" was published in 2021. Journal: J Healthc Eng.

FM data were collected from four healthy pregnant volunteers, all of whom were in a period of frequent and active FM during their gestational cycle. The average time recorded per subject was 60 minutes. During the measurement, our laboratory assistant helped the pregnant woman to wear the equipment and recorded the period during which the pregnant woman perceived the onset of FM. Before starting the experiment, the pregnant woman is asked to locate the area of the abdomen where FM is most strongly perceived and to place the device directly above that area, secured by a belt so that the sensors on either side of the device can collect the vital FM signals. A clip of the FM signal recorded based on active maternal perception is shown in Figure 7.

### 3.2. Evaluation Indicators

Real FM actively perceived by the pregnant woman is used as the standard. Evaluation indicators include true detection rate (TDR) and positive prediction value (PPV). The true detection rate represents the ratio of samples detected correctly to the total number of pieces. The positive prediction value represents the ratio of the number of positive samples detected correctly to the number of instances marked as positive in the test result.

(7) $$\begin{array}{c} \text{TDR}=100\times \frac{\text{DME}}{\text{TMF}},\\ \text{PPV}=100\times \frac{\text{DME}}{\text{DME}+\text{FD}}, \end{array}$$

where DME recognized real FM, TMF is real FM based on active maternal perception, and FD is false recognition.

## 4. Results and Discussion

The experiments were conducted using a MATLAB simulation platform to verify the performance of the proposed FM detection system. The dictionary learning database uses ZFMAD to create a complete dictionary of fetal and nonfetal features, respectively. A self-built dataset was used to test the performance of the automatic FM detection system proposed in this paper. A total of 243 segments were screened for the experiment in four pregnant women, with 39 periods of FM signals and 204 periods of non-FM signal segments. The results of the adaptive filtering-based FM signal identification are shown in Table 1. According to Table 1, it can be learned that the overall true detection rate of adaptive filtering-based FM signal identification is 92.31%, and the positive prediction value is 81.82%. Subject 3 had the best available detection, with a true detection rate of 100% and a positive prediction value of 87.5%. Although the true detection rate for subject 1 was 91.67%, the positive prediction value was only 78.85%. The reason for this may be that the artifact signal created by the random slight body movements towards the pregnant woman during the measurement is highly similar to the time-frequency characteristics of the FM signal signature, resulting in a relatively high chance of misidentification.

The article "Passive Fetal Movement Signal Detection System Based on Intelligent Sensing Technology" was published in 2021. Journal: J Healthc Eng.

The relationship curves between the sparsity and true detection rate and positive prediction value of the OMP-based algorithm for FM signal detection are shown in Figure 8. As can be seen from Figure 8, the best results in terms of true detection rate and positive prediction value of the FM signal are achieved when the sparsity *T*_0_ = 3. With sparsity greater than 9, although the positive prediction value is on an increasing trend, the true detection rate of the system decreases significantly. The ideal FM detection system would want to detect every critical FM event possible while still ensuring accuracy. Thus, the optimal parameter for the sparsity of the OMP algorithm proposed in this paper is 3. The specific results of the sparse detection of FM signals are given in Table 2.

According to Table 2, it can be observed that the overall true detection rate and positive prediction value for sparse recognition reached 89.74%. Subject 1 had the best detection, with a true detection rate and a positive prediction value of 91.67%. Subject 3 had a true detection rate of 100%, but with a positive prediction value of 87.5%; the results performed relatively poorly compared to the other three samples.

For a qualitative view of the recognition results, a graphical representation of the results is given in Figure 9.

To verify the performance of the two FM signal detection algorithms proposed in this paper, Table 3 gives a comparison of the specific results of the adaptive filtering and orthogonal matching pursuit algorithms proposed in this paper for FM recognition.  Figure 10 shows a comparison of the detection results. As observed in Table 3 and Figure 10, the TDR of the LMS was 92.31%, an increase of 2.57% compared to the TDR of the OMP algorithm, but the PPV of the LMS to detect FM was only 81.82%, a decrease of 7.92% compared to the OMP algorithm.

The article "Passive Fetal Movement Signal Detection System Based on Intelligent Sensing Technology" was published in 2021. Journal: J Healthc Eng.

To better evaluate the performance of the two FM signal detectors, it is important to consider not only the TDR and PPV of the detection but also the time to complete the detection, which reflects the computational complexity of the algorithm. The time taken for a program to run determines the efficiency of the system CPU. The longer it runs, the more CPU resources it takes up. According to Table 3, the average time taken by the LMS to finish detecting an FM signal is 5.69 s, while the OMP only takes 0.11 s on average to quickly detect the FM signal. The reason for this is that an adaptive optimization algorithm is used to adjust the filter weights and, after continuous iterative calculations, to find the appropriate weights that minimize the error between the optimal estimate and the desired signal. However, the optimal algorithm adopted is stochastic gradient descent, which requires a gradient and optimal weights for all incoming data and consumes more time in this optimization process until convergence. In contrast, the OMP algorithm introduces orthogonal features that orthogonalize all the atoms selected at each step of the decomposition, resulting in faster convergence while ensuring constant accuracy. Therefore, based on the above experimental analysis, the OMP-based FM signal detection algorithm outperforms the LMS, taking into account the true detection rate, positive prediction value, and computational cost. In this paper, the OMP-based FM signal detection algorithm is also embedded into the microprocessor system for practical performance evaluation to verify the reliability and strong robustness of the algorithm, and the experimental scenario is shown in Figure 6.

## 5. Conclusions

This paper develops a passive FM detection system based on intelligent sensing technology. Firstly, the raw FM signal acquired by the accelerometer is preprocessed using a Kalman filtering algorithm to reconstruct the FM signal in a continuous low-amplitude random noise background. The signal-to-noise ratio of the FM signal is greatly improved by constant prediction and correction. Secondly, the artifact signal is identified using an amplitude thresholding algorithm to discern the mother's characteristic artifact signal. Then, the K-SVD dictionary learning algorithm is used to learn the FM signals of 16 pregnant women from the ZFMAD public dataset to construct a complete dictionary of FM and non-FM features. The dictionary is used as the matching atom and the reference signal to identify the FM signal using orthogonal matching pursuit and adaptive filtering algorithms, respectively. Finally, a mask fusion algorithm is used to achieve FM classification. Preprocessing using Kalman filtering compensates for the traditional inability to handle unpredictable random noise signals using band-pass filtering. The shortcomings of building dictionaries from human empirical observation are addressed by machine learning methods of dictionary construction and big data analysis. The orthogonal matching pursuit algorithm and the adaptive filtering algorithm are also used to automatically match and identify FM signals and to compare their respective performances. Using four pregnant volunteers for experimental testing, the positive prediction value of the LMS-based FM signal detection algorithm was 81.82%, while the positive prediction value of the OMP algorithm reached 89.74%. Compared with the traditional TFMP, TFMF, SVM, and the recent fuzzy ARTMAP fetal movement recognition algorithm, the proposed OMP-based FM detection algorithm has improved the positive prediction value by 4.74% to 12.74%. It is worth noting that the OMP-based FM detection algorithm proposed in this paper takes only 0.11 seconds to identify FM each time. It greatly improves the operational efficiency of the system and solves the problems of the high computational cost of the traditional matching and pursuit algorithm, difficulties in running the embedded microprocessor system, and low accuracy rate. This paper also transforms the proposed algorithms into practical applications for use embedded in microprocessor systems. It was verified that the algorithm could meet the requirements of some of the mid-to-high-end microprocessor chips that exist in the market today for computing. Therefore, the FM signal recognition algorithm proposed in this paper has a high application value in micro-wearable FM monitoring devices based on acceleration sensors.

The article "Passive Fetal Movement Signal Detection System Based on Intelligent Sensing Technology" was published in 2021. Journal: J Healthc Eng.

## Figures and Tables

**Figure 1:** Flowchart of the FM detection system.

**Figure 2:** Kalman filtering results of the FM signal.

**Figure 3:** Artefactual signal of the maternal body position movement acquired by two accelerometers.

**Figure 4:** Dictionary of fetal and nonfetal movement characteristics. (a) FM dictionary. (b) Non-FM dictionary.

**Figure 5:** Flowchart of the mask fusion process.

**Figure 6:** Experiments with an FM signal acquisition and recognition system.

**Figure 7:** A fragment of an FM signal recorded by active maternal perception.

**Figure 8:** The relationship curve between accuracy and sparsity of FM signal sparse recognition.

**Figure 9:** Results of OMP-based FM detection (blue) compared with the original signal (green) and maternal perception (red). (a) Subject 1 detection result. (b) Subject 2 detection result. (c) Subject 3 detection result. (d) Subject 4 detection result.

**Figure 10:** Comparison of TDR and PPV for LMS and OMP FM signal recognition algorithms.

**Algorithm 1:** Preprocessing of FM signals.

**Algorithm 2:** FM signal sparse detection.

**Table 1:** Results of adaptive filtering-based FM recognition.

Subject	TMF	DME	FD	TDR (%)	PPV (%)
1	12	11	3	91.67	78.57
2	11	9	2	81.82	81.82
3	7	7	1	100.0	87.5
4	9	9	2	100.0	81.82
All	39	36	8	92.31	81.82

**Table 2:** Results of FM recognition based on the OMP algorithm.

Subject	TMF	DME	FD	TDR (%)	PPV (%)
1	12	11	1	91.67	91.67
2	11	9	1	81.82	90.0
3	7	7	1	100.0	87.5
4	9	8	1	88.89	88.89
All	39	35	4	89.74	89.74

**Table 3:** Comparison of FM recognition results based on LMS and OMP algorithms.

Approaches	TMF	DME	FD	TDR (%)	PPV (%)	Time (s)
LMS	39	36	8	92.31	81.82	5.69
OMP	39	35	4	89.74	89.74	0.11

## Data Availability

A part of the data used for this study is available in publicly available datasets, available online at https://doi.org/10.5281/zenodo.3544631. Another part of the data collected through the self-built system can be obtained from the corresponding author upon reasonable request.
